This article has been retracted.

# Linkages Between Knowledge Management Process and Corporate Sustainable Performance of Chinese Small and Medium Enterprises: Mediating Role of Frugal Innovation

**DOI:** 10.3389/fpsyg.2022.850820

**Published:** 2022-03-21

**Authors:** Ma Kun

**Affiliations:** Department of Philosophy, Nanjing University, Nanjing, China

**Keywords:** corporate sustainable performance, frugal innovation, knowledge management, SMEs, China

## Abstract

In the contemporary world, frugal innovation (FI) is the most discussed area to enhance corporate sustainable performance (CSP) in manufacturing firms. The knowledge management process (KMP) is also a key determinant of FI. Existing literature is limited to knowledge management (KM) and its impact on CSP. This study aims to determine the effect of the KMP (acquisition, dissemination, and application) on sustainable corporate performance with the association of FI. The survey method was used to collect data from 356 small and medium enterprises (SMEs) in China. Structure equation modeling was applied to obtain the results of collected data. Results show that all three dimensions of KM have a significant impact on CSP. Furthermore, FI also has a significant and positive impact on CSP. Results further show that FI partially mediates the relationship of the knowledge dissemination, knowledge application and sustainable corporate performance but no mediation role FI was found between knowledge acquisition and CSP. The findings of this study will provide useful insights for experts and manufacturers. It will help to understand the role of KM in their organizational behavior by being an economical manufacturing process. This study underscored the importance of the KMP to policymakers. In countries such as China that have global orders, KM is an essential determinant of FI. KM is a tool used to achieve CSP goals inside and outside of an enterprise, thus the development firms need to focus on KM.

## Introduction

A company’s success or failure depends on its knowledge. Knowledge is an intangible asset. Organizations taking the dynamic approach use it as a tool to enhance customer satisfaction and effectively compete against their competitors (Areed et al., 2021). As a result of its growing popularity in recent decades in the business world, knowledge management (KM) has been recognized as a vital element in the development of strategy, products, and services, as well as managing organizational processes. Innovation and effectiveness are enhanced by effective KM. Due to this advantage, KM has become a strategic resource for many organizations, enabling them to surpass their competitors (Lam et al., 2021). A significant component of knowledge management processes’ (KMP’s) design and development of new products and services is its management of operational processes in the current business environment. KM strategies are being adopted by organizations to achieve sustainable goals. A successful and sustainable economy relies largely on the contribution of human intellectual capital (Mohsin et al., 2021; Patel et al., 2021). In addition to helping organizations build up the capabilities required for frugal innovation (FI), KMP also assists organizations in developing a culture of corporate sustainable performance (CSP). In the development of economical products, KMP has contributed to the development of FI. KMP can, therefore, prove crucial to achieving CSP. Firms’ ability to innovate sustainably depends on their knowledge resources and capabilities (Chopra et al., 2021).

Globalization has significantly increased the demand for corporate sustainability. Environmental concerns and economic benefits are currently being focused on by organizations, but maintaining competitive edge has become a difficult task (Ayatollahi and Zeraatkar, 2020; Shahzad et al., 2020). Companies become more dynamic and agile by adopting a variety of strategies, including implementing a knowledge management process (KMP) to bolster CSP. A key component of organizational success is knowledge (Teixeira et al., 2018). Acquiring, sharing, and utilizing knowledge is being used to improve customer satisfaction and gain competitive advantages. By responding to changes with KMP, organizations improve their operations’ sustainability and competitive advantage, allowing their shareholders to feel more confident about their operations and their customers to trust them (Ceptureanu et al., 2018; Mohsin et al., 2021).

It is common to use the terms knowledge and innovation interchangeably. Studies investigating innovative processes to use knowledge as an outcome are quite common, as are studies looking at innovative processes to use knowledge as an antecedent (Durmuş-Özdemir and Abdukhoshimov, 2018). In light of this, there is a need to clarify the issue of which kind of knowledge and what kind of spill overs are more appropriate for the exact nature of innovation? The growing democratic nature of innovation has led to many of the best ideas for new products and services originating outside of well-funded corporate and government laboratories (Mirzaie et al., 2019). Ideas can originate anywhere and from anyone. In the literature, it can be found that knowledge generally originates both inside and outside a firm. Identifying, managing, sharing, leveraging, and transferring the knowledge developed internally and/or externally will support firms’ competitiveness if they adopt proper organizational and managerial practices (Brahami and Matta, 2018; Jamil et al., 2021).

Knowledge-based innovation and organizational performance are core concepts that have been studied by previous researchers to understand KMP. Although KMP and CSP have been widely discussed in the industrial world, very few studies have actually examined this relationship (Velásquez and Lara, 2021). Recently, researchers have discovered that KM and FI are connected. In their analysis of sustainable development (SD), Dost et al. (2019) cited an impact of the environmental dimension on FI. Shahzad et al. (2020) considered KM to be a powerful tool for achieving corporate SD; however, the effect of FI on KMP-CSP relationships has not been studied. Further, Nwankpa et al. (2021) emphasize the need for more research on KMP, FI, and sustainable performance.

The study findings provide manufacturers and experts with useful insights. KM plays an important role in the behavior of eco-innovative organizations because they are ecological, economic, and social corporations. KMP (acquisition, dissemination, and application) workforce growth can improve FI and CSP significantly. Providing managers with a forum for exchanging knowledge and interacting with their employees can boost their performance. The technologically advanced countries often take practical steps and invest in promoting eco-friendly technology through collaboration with other countries, who are promoting environmental concerns and CSP priorities.

The current research contributes to existing literature in numerous ways. The first contribution of this study is to fill the research gap between KMP and CSP by assessing their relationship through structural equation modeling (SEM). Furthermore, the results of this study will enable managers and experts within the organization to better integrate KM into the operations to make FI more effective. The second major contribution of this work is to shed light on a concept that is understudied in FI, augmenting CSP. In addition, this study examines Chinese industrial development, which has been less discussed in the literature. In light of CSP’s association with three primary practices, namely economic, environmental, and social sustainability, it is a good time to investigate the effects of KMPs and FIs in the workplace.

## Literature Review and Hypotheses Development

### Resource-Based View

The Resource-Based View (RBV) is a strategic management perspective originally developed with the idea of examining the relationship between organizational vulnerabilities and internal strengths and their effect on competitiveness or productivity, following a series of studies focused exclusively on industry factors determining corporate performance. Barney (2001) provides further insight into the development of sustainable competition from the perspective of company physiognomies. Physiognomies such as these are unique, inimitable, exceptional, and non-substitutive. Corporate plans and goals are significantly impacted by these tools. External resources such as these assist organizations in achieving success (Gul et al., 2021a).

In knowledge-based economies, FI and CSP are centered on KMP. In today’s fast-paced world, businesses must specialize in creativity and innovation in order to build a product that is environmentally sustainable and continuously meets clients’ and players’ demands (Velásquez and Lara, 2021). The KMP is a planned and organized initiative designed to make the most of the organization’s expertise and optimize operations. This provides mechanisms for acquiring, distributing, and efficiently utilizing organizational expertise, some of the key drivers of innovation (Abd Rahman et al., 2021; Awan et al., 2021a).

Knowledge dissemination (KD), knowledge acquisition (KA), and knowledge application (KAP) were deemed important resources for enhancing FI and CSP after popular goals (Khoa and Hoa, 2021; Naseem et al., 2022). Taking into account the ever-changing complexity of today’s market, KA is a key factor of FI in which companies learn from their interactions with various stakeholders to make sure that they advance continuously, better understanding consumer needs. In addition, the spread of awareness should be a regular practice for workers to achieve excellence (Ayatollahi and Zeraatkar, 2020; Areed et al., 2021).

Moreover, organizations use the knowledge they acquire to improve their overall processes and final products (Di Vaio et al., 2021; Gul et al., 2021b). Organizations that are knowledge-driven encourage their employees to participate in company decisions and provide dynamic solutions to organizational problems. As well as this, environmentalists and social scientists believe poor air quality and pollution are due to unsustainable product consumption. In RBV, it can be demonstrated that a company that possesses high KMPs and agile capabilities is more likely and competent to create green and sustainable products (Cheng, 2021). In addition, research shows that FI in conjunction with the KMP generates a sustainable product and has a reduced environmental, social, and ecological impact, which in turn enhances CSP (Teixeira et al., 2018; Muhammad et al., 2019).

### Knowledge Management Process and Corporate Sustainable Performance

In this study, we aim to determine if KMP specifically impacts CSP, and whether FI mediates this relationship. KM is one of the most effective ways of improving organizational innovation, which also helps discover new CSP opportunities (Awan et al., 2021b; Farza et al., 2021). A number of researchers have offered literature on the direct relationship between KMPs and innovation outputs (Gul et al., 2021c; Lam et al., 2021). Mirzaie et al. (2019) discussed that KM and varied capital are essential for creating a distinctive form of creativity. Throughout the organization, KMP and CSP work together to leverage the expertise and skills of the workforce to use green innovation tools. Research has shown that KA plays a crucial role in achieving corporate sustainability. The impact of KM on sustainable business results has also been demonstrated in recent studies (Al Mansoori et al., 2021; Areed et al., 2021). Additionally, SD has a positive effect on GI as well due to its environmental dimension. Also, FI plays an important role in corporate sustainability because the new technology and KM processes provide more versatility and improved efficiency (Gul et al., 2021d; Shahzadi et al., 2021). In addition to reducing energy demand, preventing emissions, recycling waste, and controlling the environment, advanced technologies are used to continue to enhance development. Further implementation of digital production technology contributes to the enhancement of operational productivity, which in turn impacts corporate creativity. According to Patel et al. (2021), KMP positively impacts company results through business innovation. There is no doubt that creativity and corporate sustainability are directly related, but the purpose of this study is to show that the CSP is directly influenced by KMP. In this partnership, FI, however, would have a greater impact on CSP, and it would enhance the KMP, thus making it more effective. Hence, we proposed following hypotheses:

**H1a:** Knowledge Acquisition has significant impact on corporate sustainable performance.
**H1b:** Knowledge Dissemination has significant impact on corporate sustainable performance.
**H1c:** Knowledge Application has significant impact on corporate sustainable performance.

### Knowledge Management Process and Frugal Innovation

Knowledge management process aims to provide public services and improve performance through an organized and planned approach. Chopra et al. (2021) contend that “knowledge is an intangible asset.” In fact, it can be construed as a characteristic of a company or individual that cannot be imitated. KMP also refers to the acquisition, dissemination, and implementation of business information resources in an effective manner. The use of FI as one of the key methods and experiences to achieve sustainable results is an important way to improve the system (Di Vaio et al., 2021; Zaman et al., 2022). Using existing expertise is an essential part of boosting productivity and creativity. The growth of KMP and FI is based on investing in green and natural capital. This leads to innovation based on worker skills and experience. This concept of organizational learning emphasizes the integration of corporate strategies and KM strategies to achieve FI targets (Brahami and Matta, 2018; Abbas and Kumari, 2021).

Understanding and developing new skills necessary for an organization’s productivity is the essence of learning. Most employees receive new information from their peers and co-workers within the organization. In order to assist workers in solving company problems and enhancing productivity for corporations, KAP collects information from multiple reliable sources (Sapta et al., 2021; Velásquez and Lara, 2021; Wang et al., 2021a). The previous literature on KA-FI in developed countries produced mixed findings. The relationship between KA and innovation from external markets and multiple stakeholders has been observed to be interesting. These same researchers have suggested, however, that investments in research and development can lead to more innovative performance, even if some studies find a negative correlation between KA and its performance (Rasool et al., 2019; Migdadi, 2021). There is evidence that KA has a considerable impact on developing innovative behaviors and incrementally improving performance. Khalil et al. (2021) showed that stakeholders’ collaborators’ information can influence the organizational KAP process, thereby increasing the creative output of the organization. There is little doubt that professionals and researchers around the world are interested in how information acquisition could serve as a means to achieving FI.

The dissemination of knowledge involves receiving, distributing, and transmitting knowledge among workers to boost production. The main function of it is to exchange information and to gather knowledge. Providing knowledge is the goal of sharing, whereas obtaining knowledge is the goal of collecting. By means of meetings, conferences, social networking and collaboration, these mechanisms can be shaped. Creating opportunities for learning and sharing knowledge requires intensive collaboration. A variety of studies have demonstrated how KD enhances access to information and impacts innovation. By improving operational processes and forecasts, partnerships and collaboration, corporate sustainability goals can be achieved. Despite Darroch (2005) finding that information correlates with company innovation, he showed that KD is not associated with market innovation or success in New Zealand. In addition, Zhao et al. (2022) stated that in the Chinese electronics industry, an exchange of know-how led to major advancements in FI and innovation. Based on this study, we suggest that in order to increase success rates, companies should begin by changing their information sharing behavior as their first step in making some changes. Knowledge is disbursed more widely across divisions and hierarchical levels of the company as a result of the information stream within the organization (Xu et al., 2018; Wang et al., 2021b).

Its main objective is to improve knowledge and make the company more competitive and meet consumer expectations. According to Darroch (2005), KAP is doing just that. Awareness responsiveness refers to how quickly you respond and discuss issues or potential advancements in your process or product when you are aware of consumer demands and market developments. Customer satisfaction is inextricably linked to improved consistency of service and shorter response times. Several impacts have been observed by combining KAP and GI, as shown in the previous literature. KAP has been defined by Darroch (2005) as a crucial element of organizational innovation. Another study carried out by Rezaei et al. (2020) showed that KAP is extremely important for accelerating technological advancement and efficiency. KAP and innovative green solutions are positively correlated, according to the researchers. Companies need a KAP to remain competitive in these changing times. Abubakar et al. (2019) results indicate KAP is a powerful tool for translating an organization’s knowledge into new products and processes. Furthermore, productive KAP forges a more sustainable future through creative manufacturing technologies in the interest of shareholders. There is no doubt that there is a strong connection between KAP and creativity, but it is also obvious that KAP is related to FI. Hence, we proposed following hypotheses:

**H2a:** Knowledge Acquisition has significant impact on frugal innovation.
**H2b:** Knowledge Dissemination has significant impact on frugal innovation.
**H2c:** Knowledge Application has significant impact on frugal innovation.

### Frugal Innovation and Corporate Sustainable Performance

Frugal innovation is a major way in which organizations try to minimize costs is by reducing or removing the burden of large raw material inventories. The term FI refers to the technology, goods, processes, and management systems that promote environmental conservation by reducing waste, pollution, and resource consumption (Shibin et al., 2018; Awan et al., 2021c). The isolation of method and product innovation from FI was found by Iqbal et al. (2021). New goods or procedures are improved or invented, and harmful market practices are eliminated. CSP’s new technologies and information capabilities also contribute to greater stability and efficiency, which is a key success driver. In the manufacturing of eco-friendly goods, the use of environmentally friendly technologies is advantageous to industry in two ways: first, it is economically beneficial, and second, it is competitive (Albert, 2019; Rasool et al., 2021a). In order to reduce energy consumption, emissions, waste disposal, and ecological impact, advanced technologies are being applied. A study in the past has shown that businesses need FI to use environmentally sustainable capital strategies as activities in the environment change (Shibin et al., 2018).

Rosca et al. (2018) mentioned two perspectives on economic sustainability, the first relating to financial efficiency and the second to social well-being. Due to the global economic downturn, companies and societies throughout the world are confronted with the threat of insolvency, bankruptcy, desorption, and other fiscal threats. The least expensive processes, commodities, and management can be reduced through eco-innovation, as well as R&D investment in environmental matters (Hossain, 2018; Hossain et al., 2021; Usman Shehzad et al., 2022). A number of supply-side factors are crucial to the economy and to industry efficiency, including energy cost, raw material usage, and raw material utilization. Additionally, green commodities and a healthy world have seen significant declines in manufacturing costs; however, there is no information on companies involved with green commodity innovation (Leliveld and Knorringa, 2018; Rasool et al., 2020). By minimizing industrial waste production, businesses make use of FI to increase efficiency. Researchers have also documented a positive economic impact of FI. According to the literature review, frugality innovation is critical for corporate profitability, while it does not make sense to innovate in green processes. Hence, we proposed following hypothesis:

**H3:** Frugal innovation has significant impact on corporate sustainable performance.

### Mediating Role of Frugal Innovation

When you have knowledge of technical, technological, and customer factors, it is possible to become innovative. Firms were forced to expand their innovation capabilities by fierce market competition. Innovative ideas can help businesses conduct innovation and boost their overall performance (Santos et al., 2020). ICs and knowledge can be developed through these ideas. Many companies focus solely on internal knowledge-based strategies for achieving competitive advantage in this context. Among the most important sources of internal knowledge are research and development activities, knowledge exchange and employee ideas (Dressler and Bucher, 2018). ICs can be made more effective by combining input from internal and external sources. Companies with innovative capabilities can conduct FI or make frugal products using these sources, which are more beneficial (AlMulhim, 2021).

Small and medium enterprises’ (SMEs) diverse factors can stimulate growth of FI in emerging markets. Numerous studies have shown that implementing open innovation may have a beneficial impact on encouraging FIs, especially in healthcare. Developing comprehensive knowledge of frugality is important in some regions (Gulf) and countries (e.g., Saudi Arabia) (AlMulhim, 2021). Despite the fact that there are many successful cases of small and medium Saudi Arabian businesses in anecdotal evidence, the literature rarely addresses them. The importance of innovation capabilities has been acknowledged by numerous renowned researchers. External knowledge search is defined by Dost et al. (2019) as the accessing and utilizing of external information as derived from proper sources. Innovations may be conducted by firms cooperating with external sources of knowledge to gain knowledge external to the organization (Shibin et al., 2018; Andriani et al., 2019). Academic researchers noted that collaboration patterns depend on how open a firm is to its external environment, and that different types of interaction with their external environment can produce different patterns of collaboration (Iqbal et al., 2021).

Innovating on a budget not only guarantees a strategic advantage, but also social and environmental benefits. Different core innovations concepts were developed for various market segments including environmental innovations, eco-innovations, financial innovations, and sustainable innovations (Fernandes, 2018). There are some differences between these concepts that need to be understood. Previous studies have found that sustainable engineering can be interchanged with eco-innovation, environmental innovation, and FI. Environmental innovation combines the social and eco aspects (Lei et al., 2021). However, eco-innovation considers both economic and environmental aspects. Comparatively, sustainable innovation has a strong social and moral component, and management and competition have a well-established goal. Fischer et al. (2021) suggested that we could refer to green goods and renewable processes as eco-innovation. Le (2021) described the FI as “hardware or software advancement in association with green processes and products, including advanced technology involved in saving energy, avoidance of emissions, composting, green products development, organizational environment management. Innovative application at all levels.” Innovative technologies, environmental pollution control, recycling, green product design, and ecological management are key FI priorities (AlMulhim, 2021; Hossain et al., 2021).

In order for organizations to succeed, value and sustainability must be maximized through FI. For SD to succeed, it is crucial that new concepts, products, processes, procedures, or administration systems be developed for managing environmental problems (Fischer et al., 2021). In recent years, numerous scholars have identified major factors that impact FI, such as stakeholder expectations, competitive forces and consumer desires, business ethics, and environmental awareness. In order for a company to survive, FI assessment and its aspects are considered essential (Shibin et al., 2018; Zhao et al., 2021). A competitive advantage is not the only advantage FI offers today. Legitimacy is also a precondition. Basically, “innovation” means that new products, materials, processes, administrations, and authoritative systems are more likely to give them a competitive advantage. Hence, we proposed following hypotheses:

**H4a:** Frugal Innovation mediates the relationship between knowledge acquisition and corporate sustainable performance.
**H4b:** Frugal Innovation mediates the relationship between knowledge dissemination and corporate sustainable performance.
**H4c:** Frugal Innovation mediates the relationship between knowledge application and corporate sustainable performance.

Figure 1 elaborates all the relationships.

**FIGURE 1:** Conceptual framework.

## Research Methodology

### Research Approach

Questionnaire survey method was applied in this study. To handle a large sample of a specific population this method is very appropriate and cost effective. Rasool et al. (2021b) reported that authors develop a questionnaire before the collection of data for analysis for analysis. This study also started with the development of questionnaire to collect data from respondents.

### Data Collection

We gathered data from SMEs of five Chinese largest industrial cities. A convenient sampling approach was employed (Kothari, 2004). Questionnaire was developed in English language and translation in Chinese language was also presented on questionnaire for better understanding of the responding employees. The overall sample size of this research was 356 medium and upper level management of enterprises. A total of 530 questionnaires were distributed through emails, and 370 responses were received. There were 356 appropriate replies for the final analysis, with a response rate of 67%. Valid questionnaires are selected following the survey data cleaning procedure, which involves finding and eliminating responses from respondents who either do not meet our target requirements or did not react cautiously to the questionnaire survey, such as respondents only address part of our survey; respondents provide ambiguous answers or/and select the same answer option repetitively, and respondents provide incomprehensible suggestions for open-ended questions. We employed Armstrong and Overton’s (1977) approach to determine perceived anti-reaction bias. Independent sample and Chi-square *T*-tests were conducted to analyze the initial 45 and the final 45 respondents *via* demographic factors, i.e., age and gender. The findings revealed no major variations between the two response classes (*p* > 0.05).

### Measures

The study used items established from prior research to confirm the reliability and validity of the measures. All items are evaluated through five-point Likert-type scales where “1” (strongly disagree), “3” (neutral), and “5” (strongly agree).

#### Dependent Variable

To get response about CSP we used twelve items adopted from the prior study of Bansal (2005).

#### Independent Variable

To analyze the three dimensions of KMP we used 18 items adopted from prior study of Darroch (2005). Detail of items are following:

1. Knowledge Acquisition is determined by six-items and the sample item is, “We encourage employees to take time to think about our business.”
2. Knowledge Dissemination is determined by six-items and the sample item is, “We encourage people with similar interests to work together to solve a problem.”
3. Knowledge Application is determined by six-items and the sample item is, “Information about new technological developments that might affect our business is circulated quickly.”

#### Mediating Variable

Frugal Innovation was used as mediating variable and measured with seven items adopted from the prior study of Rossetto et al. (2017) and sample item is, “We regularly search for new solutions that offer ease of use of products/services.”

### Sample Description

The demographic profile of 356 respondents, such as ownership form of the respondents, age of the organization and size of the organization, are shown in Table 1.

**TABLE 1:** Characteristics of the respondents.

Characteristics	Range	Frequency	Percentage (%)
Gender	Male	258	72.47
	Female	98	27.53
	Total	356	100.00
Age	<30 years	58	16.29
	31–35 years	85	23.87
	36–40 years	77	21.62
	41–45 years	79	22.19
	>45 years	55	15.44
	Total	356	100.00
Qualification	Bachelor	91	25.56
	Masters	81	22.75
	Post-graduate	99	27.80
	Others	85	23.87
	Total	356	100.00

### Common Method Variance

Bias due to common method variance (CMV) is a significant issue in a survey sample. This issue occurs when data is obtained from a single source (Podsakoff et al., 2003). As Harman (1976) recommends, a single-factor test was employed to determine the presence of CMV among constructs. The findings indicated that all model elements were grouped into seven constructs, with the first accounting for 34.123 percent of the total variance, less than the suggested threshold of 50% (Hair et al., 2016). Additionally, we employed Smart PLS to conduct a comprehensive collinearity investigation. According to Kock (2015) and a number of other social scientists, it is a very efficient and accurate strategy (Zafar et al., 2021). All VIF values are less than the critical limit of 5, indicating that our model does not include typical process bias (Kock, 2015).

## Results

This study employed PLS-SEM since it is the most suggested approach when the research objective is to predict and explore the dependent variables to explain the most significant variation. As a result, PLS-SEM is the most suitable predictive technique (Nitzl et al., 2016). Additionally, it can concurrently analyze measurement and structural models, making it an appropriate technique for studying complicated path model types (Hair et al., 2016). Finally, the PLS-SEM method can be used with small sample sizes yet provide reliable findings. As a result, PLS-SEM seems to be the most acceptable method for this investigation. As Cepeda-Carrion et al. (2019) has noted, the PLS-SEM approach is gaining popularity due to the potential advantages in management science (Elrehail et al., 2018). PLS-SEM seems to be adequate for this investigation in light of these arguments.

### Measurement Model Estimation

Four kinds of tests are used to validate the measurement model’s reflective constructs, including individual item reliability, internal consistency reliability, and convergent and discriminant validity. Moreover, since the research included one second-order reflective construct, namely corporate sustainable performance, the reliability, and validity of the second-order construct were also investigated. As shown in Table 2, the minimum items loading is 0.601, and the maximum is 0.898, greater than the standardized value of 0.5 (Hair et al., 2014). Internal consistency reliability was assessed through computing composite reliability (CR) and Cronbach’s alpha (Chin, 1998; Jamil et al., 2022). The researchers observed that CR is better suited for PLS-SEM. The CR value and Cronbach’s alpha values for all first and one higher order latent constructs are higher than 0.70, indicating that the measurement model was internally consistent and robust. Convergent and discriminant validity were used to determine the variable validity of the reflective measurement model. Convergent validity indicates that the degree to observe variable items assesses the same variable. The literature demonstrated that convergent validity is determined using average variance extracted (AVE) and that the AVE value for each construct must be equal to or higher than 0.50 (Hair et al., 2014). The AVE value for all first and second order construct is greater than the suggested threshold. The reliability and validity results for first and second order constructs are presented in Table 2.

**TABLE 2:** Reliability and validity analysis.

Constructs	Items	Loadings	VIF	*T* statistics	Cα	CR	AVE
Frugal innovation	FI1	0.785***	2.391	27.888	0.848	0.888	0.569
	FI2	0.777***	2.834	26.224			
	FI3	0.721***	2.130	18.889			
	FI5	0.816***	2.487	38.540			
	FI6	0.692***	1.877	17.208			
	FI7	0.728***	2.027	21.526			
Knowledge acquisition	KA1	0.794***	1.915	24.862	0.841	0.893	0.677
	KA2	0.847***	2.356	36.379			
	KA3	0.850***	2.153	40.858			
	KA4	0.799***	1.700	26.985			
Knowledge application	KAP1	0.601***	1.391	12.075	0.805	0.858	0.503
	KAP2	0.651***	1.616	13.768			
	KAP3	0.778***	1.812	27.166			
	KAP4	0.694***	1.524	20.990			
	KAP5	0.767***	1.722	34.531			
	KAP6	0.749***	1.711	24.318			
Knowledge dissemination	KD1	0.690***	1.870	20.247	0.852	0.890	0.577
	KD2	0.637***	1.738	18.090			
	KD3	0.739***	1.703	21.894			
	KD4	0.825***	2.266	34.206			
	KD5	0.814***	2.175	38.386			
	KD6	0.830***	2.403	38.588			
Corporate sustainable performance (second-order reflective construct)	ECS	0.867***	1.874	51.892	0.800	0.882	0.715
	ENS	0.812***	1.602	29.805			
	SS	0.856***	1.740	50.711			
Economic sustainability (first-order reflective construct)	ECS1	0.859***	2.253	37.532	0.884	0.920	0.742
	ECS2	0.816***	1.972	32.119			
	ECS3	0.898***	3.043	56.416			
	ECS4	0.871***	2.689	46.954			
Environmental sustainability (first-order reflective construct)	ENS1	0.713***	1.273	15.658	0.725	0.829	0.549
	ENS2	0.823***	1.692	31.964			
	ENS3	0.756***	1.526	19.990			
	ENS4	0.663***	1.271	12.441			
Social sustainability (first-order reflective construct)	SS1	0.809***	1.546	40.487	0.801	0.869	0.624
	SS2	0.807***	2.035	28.722			
	SS3	0.794***	2.005	27.940			
	SS4	0.748***	1.427	21.353			

***Significant.

Discriminant validity relates to how one construct differs statistically from another construct. Henseler et al. (2015) suggested a novel approach for assessing discriminant validity. They suggested that although the Fornell-Larcker criterion can evaluate discriminant validity efficiently, it could be unable to identify the absence of discriminant validity. Therefore, discriminant validity was analyzed using the HTMT ratio. The values of HTMT for the variables used in this study are presented in Tables 3, 4 for first and second-order constructs, respectively. According to the criteria, all variables’ HTMT values must be smaller than 0.85 (Hair et al., 2016). The results show that HTMT values for all reflective first and second-order constructs are less than 0.85, indicating the discriminant validity is established.

**TABLE 3:** Heterotrait-monotrait ratio (first order reflective measures).

	ECS	ENS	FRI	KA	KAP	KD	SS
ECS							
ENS	0.705						
FRI	0.623	0.651					
KA	0.513	0.533	0.573				
KAP	0.677	0.631	0.794	0.677			
KD	0.718	0.702	0.815	0.655	0.844		
SS	0.712	0.660	0.774	0.543	0.714	0.692	

*FI, frugal innovation; KA, knowledge acquisition; KAP, knowledge application; KD, knowledge dissemination; ECS, economic sustainability; ENS, environmental sustainability; SS, social sustainability.*

**TABLE 4:** Heterotrait-monotrait ratio (second order reflective measures).

	FRI	KA	KAP	KD	SP
FRI					
KA	0.654				
KAP	0.794	0.744			
KD	0.815	0.732	0.844		
SP	0.810	0.744	0.808	0.844	

*FI, frugal innovation; KA, knowledge acquisition; KAP, knowledge application; KD, knowledge dissemination; SP, corporate sustainable performance.*

### Structural Model

The structural model assessment phase is the second stage of PLS-SEM evaluation. The structural path model is evaluated by analyzing the model’s multicollinearity [variance inflation factor (VIF)], coefficient of determination (*R*^2^) predictive relevance (*Q*^2^), effect size (*f*^2^) and empirical significance of path coefficients, as well as the level of confidence (Hair et al., 2020). The current investigation followed the suggestions by Hair et al. (2014) for assessing the structural model and interpreting the results. Moreover, specific suggestions from Preacher and Hayes (2008) study were incorporated for mediation analysis (see Table 5).

**TABLE 5:** Effect size, coefficient of determination, and predictive relevance.

	*^f2^*		*R* ^2^	*Q* ^2^
			
	FRI	SP	Endogenous constructs	Endogenous constructs
SP			0.604	0.424
FRI		0.058	0.572	0.319
KA	0.013	0.047		
KAP	0.127	0.038		
KD	0.169	0.087		

*FI, frugal innovation; KA, knowledge acquisition; KAP, knowledge application; KD, knowledge dissemination; SP, corporate sustainable performance.*

The VIF values were analyzed in this research before the hypothesis testing to ascertain the model’s collinearity problems. According to Hair et al. (2014), if the VIF values are less than 5, there are no collinearity issues with the data. The present study’s results indicate that the components for the inner VIF have values that are much less than the suggested criterion (0.5). It demonstrates no collinearity in the data utilized in this research, confirming the model’s resilience. Additionally, our model has two endogenous components as shown in Figure 2. The *R*^2^ for FI was 0.572 (*Q*^2^ = 0.319), and CSP was 0.604 (*Q*^2^ = 0.424), which indicates that their predictors can explain 57.2 and 60.4% of the variance in the respective constructs. Moreover, the *Q*^2^ values greater than 0 indicate sufficient predictive relevance, as shown in Table 4. According to Henseler et al. (2009), an effect size of latent construct varying from 0.02, 0.15, and 0.35 is deemed minor, medium, and high, respectively. As seen in Table 5, the effect size for this study varies from small to medium, which is another evidence of the model’s robustness (Hair et al., 2016).

**FIGURE 2:** Structural model.

We next ran a bootstrapping of 5,000 subsamples to examine the proposed hypothesis. Before examining the mediation effects, we analyzed the direct relationships. Table 5 and Figure 2 illustrate the results of the direct effects. For H1a to H1c, findings reveal that KA (β = 0.103; *p* = 0.019), KD (β = 0.327; *p* < 0.001), and KAP (β = 0.223; *p* < 0.001) was significantly associated with sustainable corporate performance, which supports H1a, H1b, and H1c. Similarly, For H2a to H2c results showed that KA was insignificantly associated with FI (β = 0.061; *p* = 0.233), whereas KD (β = 0.364; *p* < 0.001) and KAP (β = 0.413; *p* < 0.001) was significantly associated with FI, indicting H2a was rejected, but H2b and H2c were accepted. Moreover, H3 results revealed that FI is positively and significantly associated with sustainable performance (β = 0.235; *p* < 0.001).

We ran the mediation analysis in Smart-PLS using the Hayes and Preacher (2010) bias-corrected bootstrapping technique with a 95% confidence interval to assess the three proposed mediating hypotheses. The results revealed that FI does not mediate the relationship between KA and sustainable corporate performance (β = 0.014; *p* < 0.277), whereas results revealed that FI significantly mediate the relationship between KD (β = 0.097; *p* < 0.001), KAP (β = 0.086; *p* < 0.002) and sustainable corporate performance (see Tables 6, 7).

**TABLE 6:** Hypotheses results.

Hypotheses	Statistical paths	Path coefficient	*T* statistics (*P*-values)	2.5–97.5%	Conclusion
Hypothesis 1a	KA → SP	0.103	2.337 (0.019)	(0.016–0.190)	Supported
Hypothesis 1b	KD → SP	0.327	5.218 (0.000)	(0.203–0.452)	Supported
Hypothesis 1c	KAP → SP	0.223	3.940 (0.000)	(0.114–0.332)	Supported
Hypothesis 2a	KA → FRI	0.061	1.192 (0.233)	(−0.040 to 0.159)	Not supported
Hypothesis 2b	KAP → FRI	0.364	5.816 (0.000)	(0.243–0.490)	Supported
Hypothesis 2c	KD → FRI	0.413	6.510 (0.000)	(0.290–0.541)	Supported
Hypothesis 3a	FRI → SP	0.235	4.106 (0.000)	(0.120–0.342)	Supported
Hypothesis 4a	KA → FRI → SP	0.014	1.088 (0.277)	(−0.009 to 0.042)	Not supported
Hypothesis 4b	KD → FRI → SP	0.097	3.946 (0.000)	(0.049–0.146)	Supported
Hypothesis 4c	KAP → FRI → SP	0.086	3.067 (0.002)	(0.036–0.145)	Supported

*FI, frugal innovation; KA, knowledge acquisition; KAP, knowledge application; KD, knowledge dissemination; SP, corporate sustainable performance.*

**TABLE 7:** Mediation results.

Mediation paths	Indirect effects	Total effects	VAF (%)	Results
KA → FRI → SP	0.014	0.117	12.221	No meditation
KD → FRI → SP	0.097	0.424	22.913	Partial meditation
KAP → FRI → SP	0.086	0.309	27.697	Partial meditation

Moreover, the variance accounted for (VAF) method was employed to assess the mediation effect of FI in mediating the relationship between KA, KD, KAP, and CSP. As a general rule, VAF values more than 80, 20–80%, and less than 20% are termed full mediation, partial mediation, and no mediation, respectively. Table 6 shows that the VAF value is 12.221, 22.913, and 27.697%, respectively. These results reveal that FI does not mediate the relationship between KA and sustainable corporate performance, but partially mediates the relationship between KD, KAP, and sustainable performance.

## Discussion and Conclusion

In order to determine what role FI plays in overall process improvements for RBV (Barney, 2001) manufacturers, this study examined how KMP strengthens FI. The innovation process has led to a drop in competitiveness in these industries. According to the current study, KMP contributes to FI, and FI contributes to CSP. Furthermore, the KMP dimensions (KA, KD, and KAP) confirmed the original study’s findings across a broader range of variables, demonstrating a beneficial interaction with FI. By using specialized expertise, any problem can be viewed differently, and, for instance, financial capability growth, employee capabilities, and customer demands can be considered.

Nwankpa et al. (2021) argued that there was no relationship between KA and performance of organizations in their previous study. This research contradicts their findings. The results of previous research indicate that KD is positively related to FI. Let’s say that organizations are able to exchange expertise amongst all employees. Thus, they improve performance, including operational, financial, and non-economic aspects, while coordinating multiple stakeholders to achieve eco-innovation. Additionally, creative success and expertise can be enhanced through KD. In contrast to Darroch (2005) prior research, our findings indicate that KD is positively correlated with firm success. We found that introverted workers disseminate less knowledge. Recently, several studies have found similar results (Mirzaie et al., 2019; Shahzad et al., 2020; Areed et al., 2021). In addition, KAP and FI appear to be strongly linked. The companies must be able to adapt already acquired information quickly and easily to achieve full customer loyalty. As a result of advanced technologies and products reliant on KAP, Darroch (2005) suggests that business operations could produce green goods more easily. The FI is seen as one of the major drivers of corporate sustainability, culminating in the CSP, according to previous research (Di Vaio et al., 2021). Corporate sustainability is largely driven by FI, which is viewed as a key driver of CSP, ultimately resulting in corporate sustainability. This study reveals that the effect of FI on CSP measurements is both significant and optimistic.

Knowledge management process/corporate sustainable performance interact *via* FI according to results of the mediation analysis. It is essential to better understand FI’s critical role in mediating KMP and CSP based on research in the past. Therefore, the current study’s findings strengthened FI’s mediating position and established the possibility that CSP and KMP are partly mediated (Migdadi, 2021). A mild relationship between FI and CSP was also examined and it was found that the relationship is positive. The interactions with FI and CSP with KMP were, however, remarkably negligible. This study is unique, and an important contribution to literature.

### Practical Implications

Firstly, the study findings provide manufacturers and experts with useful insights. KM plays an important role in the behavior of eco-innovative organizations because they are ecological, economic, and social corporations. KMP (acquisition, dissemination, and application) workforce growth can improve FI and CSP significantly.

In addition, this study underscored the importance of the KMP to policymakers. Companies should take an active role in training their managers and building a successful organization. In countries such as China that have global orders, KM is an essential determinant of FI. KM is a tool used to achieve CSP goals inside and outside of an enterprise, thus the development firms need to focus on KM. Providing managers with a forum for exchanging knowledge and interacting with their employees can boost their performance. The technologically advanced countries often take practical steps and invest in promoting eco-friendly technology through collaboration with other countries, who are promoting environmental concerns and CSP priorities.

### Limitations and Future Research Direction

A limited time and budget limit this study, which could hamper potential researchers. In addition, the study was limited to one country and the manufacturing sector. A more detailed study should be conducted by extending the scope of this research to many regions. Other areas may also be considered when comparing the findings of this research. This study could also be applied to a specific business sector, which will make it more generalizable. Although this study offers a roadmap for uncertified businesses, future research will also provide knowledge-based insight into uncertified organizations on an organizational and industry level. Prospective or experimental research is also recommended for obtaining more conclusive results in the future. Further, employees’ personality attributes, such as their complex and absorbent qualities, may be considered as moderating factors. In the successful KM phase, absorbent capacity and personality characteristics (extraverted versus introverted) are necessary for the acquisition and sharing of information.

## Data Availability Statement

The raw data supporting the conclusions of this article will be made available by the authors, without undue reservation.

## Author Contributions

The author confirms being the sole contributor of this work and has approved it for publication.

## Conflict of Interest

The author declares that the research was conducted in the absence of any commercial or financial relationships that could be construed as a potential conflict of interest.

## Publisher’s Note

All claims expressed in this article are solely those of the authors and do not necessarily represent those of their affiliated organizations, or those of the publisher, the editors and the reviewers. Any product that may be evaluated in this article, or claim that may be made by its manufacturer, is not guaranteed or endorsed by the publisher.

## Appendix

**Appendix 1:** Questionnaire.

**Knowledge management process**
***Knowledge acquisition***
We survey employees regularly to access their attitude toward work
Managers frequently try to find out employees “true feelings about job”
We have regular staff appraisals in which we discuss the needs of our employees
Employees are encouraged to attend training seminars and conferences
We encourage employees to take time to think about our business
We have regular meetings with employees
***Knowledge dissemination***
Marketing people in our organization frequently spend their time discussing customer’s future needs with people in technical department
We encourage people with similar interests to work together to solve a problem
We frequently use techniques such as quality circles in our organization
We often use video conferencing within our organization
We frequently update policy and procedure manuals
Our organization actively encourages mentoring or coaching
***Knowledge application***
We usually respond to changes in our customer’s product or service need
We are quick to respond customer’s complaints
Our organization seems to be able to implement marketing plans effectively
Information about new technological developments that might affect our business is circulated quickly
When something important happens to a competitor the whole organization knows about it quickly
We frequently change our technical strategies
***Frugal innovation***
We regularly search for new solutions that offer ease of use of products/services
We use the fewest amount of materials to comprise the product for conducting the product development or design
We would circumspectly deliberate whether the product is easy to recycle, reuse, and decompose for conducting the product development or design
The manufacturing process of the company reduces the consumption of water, electricity, coal, or oil
We regularly improve the durability of the products/services
The manufacturing process of the company effectively reduces the emission of hazardous substances or waste
The manufacturing process of the company reduces the use of raw materials
**Corporate sustainable performance**
***Environmental sustainability***
Mined/manufactured products that have a less environmentally harmful impact than in previous years or than its competitors
Chose inputs from sources that are remediated or replenished
Reduced waste by streamlining processes
Handled or stored toxic waste responsibly
***Economic sustainability***
Worked with government officials to protect the company’s interests
Reduced costs of inputs for same level of outputs
Reduced costs for waste management for same level of outputs
Solid waste product for revenue
***Social sustainability***
Considered interests of stakeholders in investment decisions by creating a formal dialogue
Improved employee or community health and safety
Protected claims and rights of aboriginal peoples or local community
Showed concern for the visual aspects of the firm’s facilities and operations
